The article "Molecular characterization of forest soil based Paenibacillus elgii and optimization of various culture conditions for its improved antimicrobial activity" was retracted in 2017. Reason: compromised peer review.

# Molecular characterization of forest soil based *Paenibacillus elgii* and optimization of various culture conditions for its improved antimicrobial activity

**DOI:** 10.3389/fmicb.2015.01167

**Published:** 2015-10-21

**Authors:** S. N. Kumar, Jubi Jacob, U. R. Reshma, R. O. Rajesh, B. S. D. Kumar

**Affiliations:** Agroprocessing and Natural Products Division, Council of Scientific and Industrial Research – National Institute for Interdisciplinary Science and Technology, Thiruvananthapuram, India

**Keywords:** *Paenibacillus elgii*, cultural condition, antimicrobial metabolites, improvement, carbon source

## Abstract

Microorganisms have provided a bounty of bioactive secondary metabolites with very exciting biological activities such as antibacterial, antifungal antiviral, and anticancer, etc. The present study aims at the optimization of culture conditions for improved antimicrobial production of *Paenibacillus elgii* obtained from Wayanad forest of Western Ghats region of Kerala, India. A bacterial strain isolated from the Western Ghats forest soil of Wayanad, Kerala, India was identified as *P. elgii* by 16S rRNA gene sequencing. *P. elgii* recorded significant board spectrum activity against all human and plant pathogenic microorganism tested except *Candida albicans*. It has been well known that even minor variations in the fermentation medium may impact not only the quantity of desired bioactive metabolites but also the general metabolic profile of the producing microorganisms. Thus, further studies were carried out to assess the impact of medium components on the antimicrobial production of *P. elgii* and to optimize an ideal fermentation medium to maximize its antimicrobial production. Out of three media [nutrient broth (NA), Luria broth (LB) and Trypticase soy broth (TSB)] used for fermentation, TSB medium recorded significant activity. Glucose and meat peptone were identified as the best carbon and nitrogen sources, which significantly affected the antibiotic production when supplemented with TSB medium. Next the effect of various fermentation conditions such as temperature, pH, and incubation time on the production of antimicrobial compounds was studied on TSB + glucose + meat peptone and an initial pH of 7 and a temperature of 30°C for 3 days were found to be optimum for maximum antimicrobial production. The results indicate that medium composition in the fermentation media along with cultural parameters plays a vital role in the enhanced production of antimicrobial substances.

## Introduction

During the last few decades, there has been a concomitant rise in the occurrence of multidrug-resistant (MDR) pathogens that have caused serious problems to humans worldwide (Ajesh et al., 2013). The growing tendency of various microbial infections, the rapid emergence of MDR to current antibiotics and quick evolution through mutation are of a significant threat to the control of various microbial infections (Roy et al., 2013). Unfortunately, few new antibiotics have been developed precisely for treating MDR microbes in recent years (Vaara et al., 2010; Velkov et al., 2010). The development of novel antibiotics cannot keep up with the evolution of antimicrobial resistance of bacteria against various drugs. Thus, there is a great need for discovering and developing new antimicrobial drugs to combat the drug-resistant pathogens. The natural compounds with medicinal importance are primarily produced from the primary and secondary metabolism of various microorganisms and plants. Interestingly, microbial based natural compounds have made an incredible input to the antimicrobial drug discovery and its development process over past seven decades (Jose and Jebakumar, 2013). Microbial based natural compounds are the origin of most of the antimicrobial drugs available on the market today. But now a day there is a disturbing shortage of novel antimicrobial drugs currently under development in the pharmaceutical industry. Still, these natural compounds from microbial sources remain as the most talented source of many new antibiotics, although new tactics are still required to improve the competence of the current drug discovery process.

The article "Molecular characterization of forest soil based Paenibacillus elgii and optimization of various culture conditions for its improved antimicrobial activity" was retracted in 2017. Reason: compromised peer review.

Production of bioactive secondary metabolites by microorganisms significantly depends on the species and strains of microorganisms, its nutritional, and cultural conditions (Jose et al., 2011; Wang et al., 2011). Minor variations in the fermentation media composition play a profound role in quantity and quality of secondary metabolites production (Wang et al., 2011). Hence, optimization of the fermentation medium is very much essential to confirm enhanced production of desired metabolites. Improving the antibiotic production is the prerequisite to achieving adequate antibiotic yield for evaluating its potential and novelty. The antibiotic producing ability of the microorganism is not a static property and it is highly influenced by culture conditions and media components used (Hassan et al., 2001; Gunnarsson et al., 2003). Therefore, designing a suitable fermentation medium and conditions has vital importance in improving the antibiotic yield and easing the cost of production (Wang et al., 2008; Feng et al., 2011). Moreover designing an appropriate fermentation system for a good producer strains require a series of trials like selection of basal medium, selection of best carbon and nitrogen sources, optimization of the physical parameters, screening for each medium components which have significant impact on production of particular compound, and optimization of influencing medium components (Wang et al., 2011). However, studies on the development of ideal production medium and culture conditions for the consistent production of antibiotics from *Paenibacillus elgii* remain scarce in the literature. Thus, the present paper is the first report on the optimization of the culture conditions for the maximum production of antimicrobial metabolites by *P. elgii.*

The article "Molecular characterization of forest soil based Paenibacillus elgii and optimization of various culture conditions for its improved antimicrobial activity" was retracted in 2017. Reason: compromised peer review.

## Materials and Methods

### Strain and Its Maintenance

The *Paenibacillus* strain used in this work designated as *P. elgii* NIISTB523 was isolated from the forest soil of Western Ghats region of Wayanad, Kerala, India and has the ability of producing antimicrobial metabolites against a wide range of bacteria. Briefly, soil samples (approximately 10 g) were collected in a sterile polythene bag using a sterile spatula. 1 g of the soil samples were dissolved in 10 ml of sterile distilled water to make soil suspensions. Portions of the suspension were inoculated on the nutrient agar and incubated at 37°C for 24 h. After which *P. elgii* colonies showing a clear zone of inhibition were isolated. After isolation, the *P. elgii* was maintained on nutrient agar (NA) medium at 30°C.

### Molecular Identification of the Organism

Genomic DNA was isolated from the bacterium using DNeasy^®^ Blood and Tissue Kit (Qiagen) following manufacturer’s instructions. A portion of the culture was transferred to 180 μl of ATL buffer and followed by the addition of proteinase K (20 μl) and incubated at 56°C in a water bath until the cells were fully lysed. After lysis, RNase A (5 μl, 100 mg/ml) was added and incubated for 5 min at room temperature. Then 200 μl of AL buffer and 200 μl of ethanol (100%) were added followed by thorough mixing by vortexing. After that, the mixture was transferred into DNeasy Mini spin column placed in a 2 ml collection tube and centrifuged at 8000 rpm for 1 min. After centrifugation the DNeasy mini spin column was shifted to a new 2 ml tube and washed with 500 μl of the AW1 buffer. Wash step was repeated using the AW2 buffer. After through washing the DNeasy mini spin column was placed in a clean 1.5 ml tube and DNA was eluted out using 50 μl of AE buffer.

The quality of the isolated DNA was checked using agarose gel electrophoresis. The complete 16S rRNA fragment was prepared by PCR and the amplification reactions were carried out in a 20 μl reaction volume which contained 1X PCR buffer (100 mM Tris-HCl, pH 8.3; 500 mM KCl), 0.2 mM each dNTPs (dATP, dGTP, dCTP, and dTTP), 2.5 mM MgCl_2_, 1 unit of AmpliTaq Gold DNA polymerase enzyme, 0.1 mg/ml BSA, 4% DMSO, 5 pM of forward (16S-UP-F-CGAATTCGTCGACAACAGAGTTTGATCCTGGCTCAG) and reverse (16S-UP-R-CCCGGGATCCAAGCTTACGGCTACCTTGTTACGACTT) primers and FTA disk as template. The PCR amplification was carried out in a PCR thermal cycler (GeneAmp PCR System 9700, Applied Biosystems, USA). PCR conditions consisted of an initial denaturation step at 94°C for 5 min followed by 35 amplification cycles of 94°C for 1 min, 55°C for 45 s, and 72°C for 1 min. Sequencing reaction was done in a PCR thermal cycler (Gene Amp PCR System 9700, Applied Biosystems, USA) using the Big Dye Terminator v3.1 Cycle Sequencing Kit (Applied Biosystems, USA) following manufacturers protocol. The sequence quality was checked using Sequence Scanner Software v1 (Applied Biosystems). Sequence alignment and required editing of the obtained sequences were carried out using Geneious Pro v5.6 (Drummond et al., 2012).

The article "Molecular characterization of forest soil based Paenibacillus elgii and optimization of various culture conditions for its improved antimicrobial activity" was retracted in 2017. Reason: compromised peer review.

### Phylogenetic Analysis

The nucleotide sequence obtained was finally processed to remove low-quality reads, transformed into consensus sequences with Geneious Pro software version 5.6. The resulted high-quality sequences were analyzed with BLASTn (NCBI) to confirm the final authenticity of the isolated bacterium. The DNA sequences of closely related species and genus were downloaded from the NCBI Genbank database and phylogenetic conductions was carried out with the MEGA version 5 program. Then the sequences were aligned using the ClustalW and were then analyzed to determine the relationships between other closely related isolates by the neighbor-joining method using the Maximum Composite Likelihood model. Bootstrap values were produced using 1500 replicates.

### Test Pathogens

#### Bacteria

Gram-positive bacteria: *Bacillus subtilis* MTCC 2756, *Staphylococcus aureus* MTCC 902, *S. epidermidis* MTCC 435 and *S. simulans* MTCC 3610; Gram-negative bacteria: *Escherichia coli* MTCC 2622, *Klebsiella pneumoniae* MTCC 109, *Proteus mirabilis* MTCC 425, *Vibrio cholerae* MTCC 3905, *Pseudomonas aeruginosa* MTCC 2642, and *Salmonella typhi* MTCC 3216.

#### Fungi

Medically important fungi: *Aspergillus flavus* MTCC 183, and *Trichophyton rubrum* MTCC 296, *Candida albicans* MTCC 277 and agriculturally important fungi: *A. niger* MTCC 282, *A. fumigatus* MTCC 3376, *A. tubingensis* MTCC 2425, *Fusarium oxysporum* MTCC 284, *Rhizoctonia solani* MTCC 4634, *Colletotrichum gloeosporioides* MTCC 10183, and *Penicillium expansum* MTCC 2006. All the test microorganisms were procured from Microbial Type Culture Collection Centre (MTCC), IMTECH, Chandigarh, India. The test bacteria were maintained on nutrient agar slants and test fungi were maintained on potato dextrose agar slants.

The article "Molecular characterization of forest soil based Paenibacillus elgii and optimization of various culture conditions for its improved antimicrobial activity" was retracted in 2017. Reason: compromised peer review.

### *In Vitro* Antibiosis of *P. elgii*

#### Against Bacteria

The agar overlay method was used for the examination of intact *P. elgii* inhibitory effect against test bacterial pathogens. In this method, the plate containing the 2 days old culture of *P. elgii* strain was overlaid with the top nutrient agar (Hi-media, Mumbai, India) which contains the test bacterial strains. The inhibitory effect was evaluated after 18 h incubation at 37°C and the results were evaluated by the measurement of inhibition zone of diameter expressed in millimeter (mm).

#### Against Fungi

The dual culture technique was employed to find out the inhibitory activity of *P. elgii* against filamentous fungi (*F. oxysporum*, *R. solani*, and *C. gloeosporioides*) on PDA agar medium (Naing et al., 2014). The dual cultured plates after treatment were then incubated for 5 days at 28°C. The agar overlay method with fungal spores was employed for detecting the activity of *P. eligii* against spore forming test fungi. *P. elgii* were inoculated as spot on nutrient agar plates and incubated at 30°C for 48 h. Then the plates were overlaid with potato dextrose agar containing 1 × 10^6^ spores of each fungus per ml. After 48–72 h of incubation at 30°C, the inhibition zone was measured. For *Candida* sp. agar overlay method, as described above for the bacteria, were adopted.

### Standardization of Optimal Fermentation Medium for Maximum Antimicrobial Production

Three different standard media such as nutrient broth (NA), Luria broth (LB), and Trypticase soy broth (TSB) were used in comparative studies to find the best fermentation medium for antimicrobial production. Five microliter of the seed culture was transferred into 100 ml of different sterile medium in 250 ml flask. The flasks were incubated in the dark at 150 rpm for 72 h at 30°C on a rotary shaker. After incubation, the culture media were then centrifuged (10,000 *g*, 20 min, 4°C) followed by filtration through a 0.45 μm filter, to obtain cell free culture filtrate.

### Preparation of Crude Organic Extract

The cell free culture filtrate was neutralized with concentrated HCl and extracted with an equal volume of ethyl acetate thrice. The ethyl acetate extracts were combined, dried over anhydrous sodium sulfate, and concentrated using a rotary flash evaporator at 40°C to obtain the crude extract.

### Assay of Antibiotic Activity of Crude Extract (Agar Disk Diffusion Assay)

Antibiotic activity of the crude extracts was measured by agar disk diffusion assay. Briefly, 0.1 ml containing 10^6^–10^7^ CFU/ml of test bacteria was swabbed into Mueller Hinton Agar (MHA) plate. The crude extract (100 μl) following microfiltration using a 0.22 μm syringe microfilter, were loaded on 6 mm sterile disk filters (Whatman 3-mm paper, Hi-media) and air dried. After 2 h incubation at room temperature, the dried disks were placed on the MHA plate and incubated at 37°C for 18 h to determine the diameter of zone of inhibition and expressed in millimeter (mm; Wang et al., 2011). The experiment was performed in triplicate.

The article "Molecular characterization of forest soil based Paenibacillus elgii and optimization of various culture conditions for its improved antimicrobial activity" was retracted in 2017. Reason: compromised peer review.

### Selection of Best Carbon and Nitrogen Sources for Maximum Antimicrobial Production

In order to examine the effect of the different carbon and nitrogen sources on the antimicrobial production of the potential microbe, the best nutrient medium for antimicrobial production was employed as an original medium for the following optimization studies. In this study, TSB media was used as original medium (recorded maximum activity in the initial standardization studies). One percentage (1%) of eight simple and complex carbon (glucose, maltose, starch, fructose, lactose, glycerol, mannitol, and sucrose) and 12 nitrogen (peptone, yeast extract, meat peptone, soyabean meal, beef extract, meat extract, malt extract, biopeptone, meat infusion, potassium nitrate, urea, ammonium sulfate) sources were used independently instead of the corresponding carbon and nitrogen sources in the original best nutrient medium while other medium components were kept constant at its original concentration. The bacterial fermentation was carried out for 72 h of incubation at 28°C with shaking at 150 rpm and the crude extract was isolated according to the method mentioned earlier. The antimicrobial activity of the crude extract was determined by agar disk diffusion assay.

### Impact of Temperature, pH and Incubation Period on the Enhanced Production of Antimicrobial Compounds

The outcome of culture condition on the production of the enhanced antimicrobial production was studied on TSB supplemented with 1% of glucose and meat peptone against *K. pneumoniae* (recorded significant activity in initial standardization studies). The impact of temperature on growth and production of antimicrobial compounds was investigated on TSB + glucose + meat peptone at different temperatures (20, 22, 25, 28, 30, 32, 35, 38, and 40°C) at pH 7. Ten ml suspension of the bacterial isolate was inoculated into 100 ml of TSB + glucose + meat peptone in 250 ml Erlenmeyer flask and incubated in a shaking incubator upheld at 150 rpm for 4 days at 28°C. The antimicrobial activity was assessed against *K. pneumoniae* by agar disk diffusion assay as mentioned above. Likewise, the impact of pH on the antimicrobial compounds production was studied at various pH range (4–9) using TSB + glucose + meat peptone by incubating at 28°C for 4 days. The impact of incubation period on the antimicrobial production was also studied in the similar way as above by incubating for various days (1–7) at 28°C using TSB + glucose + meat peptone at pH 7.

The article "Molecular characterization of forest soil based Paenibacillus elgii and optimization of various culture conditions for its improved antimicrobial activity" was retracted in 2017. Reason: compromised peer review.

### Antibacterial Activity of TSB + Glucose + Meat Peptone in the Best Ideal Condition

TSB + glucose + meat peptone with an initial pH of 7 was prepared and the fermentation was carried for 3 days at 30°C (best ideal condition that was already standardized) under shaking (150 rpm). The crude extract was isolated after fermentation as described earlier and the antibacterial activity was carried out using agar disk diffusion assay against all test bacteria. Ciprofloxacin was used as reference antibiotic.

### Statistical Analysis

The statistical analyses of the data were achieved using SPSS (Version 17.0; SPSS, Inc., Chicago, IL, USA). Antimicrobial results were reported as mean ± standard deviations. Duncans multiple range tests (DMRT) was done to compare that the sample means were significantly different from each other at a significant level of *P* > 0.05.

## Results

### 16S rRNA Sequencing and Phylogenetic Analysis of the Strain

The isolate NIISTB523 was identified as *P. elgii* based on 16S rRNA gene sequencing. PCR amplification yielded ∼1500 bp amplicon. Blast analysis showed greater than 99% similarity to *P. elgii* sequences available in the NCBI Genbank database and thus the isolates were finally acknowledged as *P. elgii.*

Sequence data for the 16S rRNA gene of *P. elgii* was finally deposited in the NCBI GenBank nucleotide database under the Ac. No. (KM288623). The phylogenetic tree clearly showed the relationships of the isolates used in the analysis. The present bacterium (*P. elgii*) was successfully grouped along with other *P. elgii* isolates obtained from the NCBI Genbank database confirming the genuineness of the isolate (**Figure 1**).

**FIGURE 1:** **(A)** *Paenibacillus elgii* isolate was grown on nutrient agar plates. **(B)** Neighbor joining Phylogenetic tree showing the position of isolate *P. elgii* with other species of the genus *Paenibacillus* sp. and related taxa based on 16S rDNA gene sequences. Bootstrap values (expressed as percentages of 1000 replications) are indicated.

### *In Vitro* Antibiosis of the *P. elgii* Against the Test Microbes

*In vitro* antibiosis of the *P. elgii* against the test bacteria was shown in **Table 1**. *P. elgii* displayed significant antimicrobial activity against all test bacteria and the best activity was recorded against *B. cereus* (55 mm) and *S. epidermidis* (52 mm; **Table 1** and **Figure 2**). *P. elgii* also recorded significant *in vitro* antifungal activity against all the test fungi except *C. albicans* and significant activity was recorded against *P. expansum* (31 mm; **Table 1** and **Figure 3**).

The article "Molecular characterization of forest soil based Paenibacillus elgii and optimization of various culture conditions for its improved antimicrobial activity" was retracted in 2017. Reason: compromised peer review.

**Table 1:** *In vitro* antibiosis of the *Paenibacillus elgii* against test microbes.

Test bacteria	Zone of Inhibition (mm)	Test fungi	Zone of Inhibition (mm)
*B. cereus*	55 ± 3.25	*A. flavus*	17 ± 1.27
*B. subtilis*	27 ± 2.15	*C. albicans*	-
*S. aureus*	41 ± 1.75	*T. rubrum*	25 ± 0
*S. epidermis*	52 ± 2.75	*A. niger*	22 ± 0.57
*S. simulans*	47 ± 2.12	*A. fumigatus*	29 ± 1.52
*E. coli*	48 ± 3.15	*A. tubengensis*	20 ± 0.77
*K. pneumoniae*	40 ± 1.85	*F. oxysporum*	15 ± 0.52
*P. mirabilis*	25 ± 0	*R. solani*	14 ± 1.77
*P. aeruginosa*	44 ± 1	*C. gloeosporioides*	17 ± 0.77
*S. typhi*	35 ± 1.85	*P. expansum*	31 ± 1


*-, Recorded no activity.*

**FIGURE 2:** ***In vitro* antibiosis of *P. elgii* against test bacteria**.

**FIGURE 3:** ***In vitro* antibiosis of *P. elgii* against test fungi. (A)** Sporulation fungi and **(B)** filamentous fungi.

### Standardization of Optimal Fermentation Medium for Maximum Antimicrobial Production

#### Yield of Crude Extract in Standard Media

The maximum yield was recorded for TSB (567 mg/L), followed by LB (423 mg/L), and nutrient broth (235 mg/L).

#### Antibacterial Activity of Crude Extract

The antibacterial activity of crude extracts from standard media is shown in **Table 2**. TSB medium recorded maximum activity. The most sensitive test bacteria to the TSB crude extract was *B. cereus* (27 mm).

**Table 2:** Antimicrobial activity of crude extract.

Test microbes	Zone of inhibition (mm)		
	
	TSB	LB	NB
*B. cereus*	27 ± 0	21 ± 0	11 ± 0
*B. subtilis*	23 ± 1.15	16 ± 1	13 ± 0
*S. aureus*	20 ± 1.72	17 ± 1.12	-
*S. epidermis*	25 ± 0.52	15 ± 1.77	12 ± 0
*S. simulans*	23 ± 1	20 ± 1.12	15 ± 1
*E. coli*	21 ± 1	12 ± 0	13 ± 1.72
*K. pneumoniae*	24 ± 0	14 ± 1.75	12 ± 2.20
*P. mirabilis*	20 ± 2.25	13 ± 0	-
*P. aeruginosa*	21 ± 1.75	11 ± 1.12	-
*S. typhi*	24 ± 1.12	17 ± 1	-


*-, Recorded no activity.*

### Selection of Best Carbon and Nitrogen Sources for Maximum Antimicrobial Production

The yield of crude extract from TSB supplemented with different carbon and nitrogen sources are shown in **Figure 4**. In case of TSB supplemented with different carbon sources, the highest yield was recorded by TSB + glucose, followed by TSB + fructose (**Figure 4A**). Whereas in the case of TSB supplemented with different nitrogen sources, the highest yield was recorded by TSB + meat peptone (**Figure 4B**).

**FIGURE 4:** **Yield of crude extract in TBS media supplemented with different carbon sources and nitrogen sources. (A)** Carbon sources and **(B)** nitrogen sources. Different letters in the superscript were significantly different according to Duncan’s multiple range test (*p* < 0.05).

The article "Molecular characterization of forest soil based Paenibacillus elgii and optimization of various culture conditions for its improved antimicrobial activity" was retracted in 2017. Reason: compromised peer review.

In case of the antimicrobial activity of crude extract from different carbon sources, significant activity was recorded by TSB + glucose (**Table 3** and **Figure 5**), followed by TSB + glycerol. Similarly in case of TSB supplied with nitrogen sources, significant activity was recorded by TSB + meat peptone (**Table 4** and **Figure 5**), followed TSB + yeast extract. *K. pneumoniae* was the most sensitive organism to the extract (**Tables 3** and **4**). All the combination recorded antimicrobial activity. But certain combination recorded lower activity than the TSB medium alone.

**Table 3:** Antimicrobial activity of crude extract in TBS media supplemented with different carbon sources.

Test microbes	Zone of inhibition (mm)							
	
	Sta	Mal	Glu	Fru	Lac	Gly	Man	Suc
*B. subtilis*	15 ± 1	13 ± 1.12	27 ± 0	22 ± 1.11	11 ± 0.52	21 ± 0.52	12 ± 0.57	22 ± 1.12
*S. aureus*	16 ± 1	19 ± 052	23 ± 0	16 ± 0.77	14 ± 0	22 ± 0	14 ± 0	21 ± 0
*S. epidermis*	14 ± 0	15 ± 1	28 ± 1	23 ± 1.12	15 ± 1.12	24 ± 1	13 ± 0	19 ± 1.56
*S. simulans*	16 ± 1.12	21 ± 1	27 ± 1.15	23 ± 1.57	13 ± 0.77	25 ± 1.27	13 ± 1	20 ± 0
*B. cereus*	19 ± 0.77	22 ± 0	29 ± 0.52	21 ± 2.17	17 ± 1	21 ± 1.56	12 ± 1	18 ± 1
*E. coli*	20 ± 2.21	14 ± 0	26 ± 0.77	25 ± 2.72	19 ± 1	26 ± 2.72	16 ± 1.12	17 ± 1.72
***K. pneumoniae***	21 ± 0	19 ± 1.12	**31 ± 1.17**	21 ± 1.77	21 ± 0	19 ± 1.77	15 ± 0.57	15 ± 1.77
*P. mirabilis*	23 ± 1	23 ± 1.77	26 ± 1.72	17 ± 0.52	14 ± 1.12	18 ± 1.52	19 ± 0.52	19 ± 1.52
*P. aeruginosa*	18 ± 0.77	21 ± 1.52	24 ± 0.77	18 ± 0	17 ± 1.77	23 ± 0.57	21 ± 1.52	21 ± 0.57
*S. typhi*	19 ± 0.52	22 ± 2.12	25 ± 0.52	19 ± 1	15 ± 0.22	21 ± 0.52	20 ± 1.77	18 ± 2.12


*Bold indicated the best activity displayed by glucose against K. pneumoniae.*

**FIGURE 5:** **Antibacterial activity of TSB medium and modified media**.

**Table 4:** Antimicrobial activity of crude extract in TBS media supplemented with different nitrogen sources.

Test microbes	Zone of inhibition (mm)											
	
	Peptone	Yeast extract	Meat peptone	Soyabean meal	Beef extract	Meat extract	Malt extract	Biopeptone	Meat infusion	Potassium nitrate	Urea	Ammonium sulfate
*B. cereus*	20 ± 0.27	24 ± 1.57	29 ± 0	21 ± 1	20 ± 1.56	22 ± 0.56	15 ± 2.77	21 ± 1.77	21 ± 0.77	13 ± 1.25	16 ± 1.77	13 ± 2.21
*B. subtilis*	18 ± 1.56	21 ± 0.56	30 ± 1.56	22 ± 1	21 ± 1.52	21 ± 1.12	13 ± 0.77	18 ± 0.56	21 ± 0	12 ± 0	11 ± 0.77	14 ± 0.52
*S. aureus*	19 ± 1	21 ± 1.72	25 ± 0.52	19 ± 0	22 ± 1.12	22 ± 1.72	15 ± 0.52	20 ± 0.57	14 ± 0	12 ± 0.56	14 ± 1	19 ± 0.77
*S. epidermis*	19 ± 0	17 ± 0.52	30 ± 0.56	20 ± 0.52	23 ± 2.12	23 ± 1.121	16 ± 1	19 ± 1.77	17 ± 0.52	15 ± 1.15	15 ± 0	12 ± 1.52
*S. simulans*	21 ± 1.22	23 ± 1	31 ± 1.56	21 ± 0.22	24 ± 0.56	24 ± 0.56	17 ± 1	21 ± 2.52	19 ± 0.56	17 ± 1.72	14 ± 1.12	17 ± 1.57
*E. coli*	22 ± 1.56	21 ± 1	26 ± 1.72	15 ± 0.77	21 ± 0.57	21 ± 0.75	18 ± 0	22 ± 2.12	20 ± 1.71	14 ± 0.77	17 ± 1.52	14 ± 2.52
***K. pneumoniae***	20 ± 1.77	19 ± 0.57	**33 ± 1.77**	17 ± 0.72	21 ± 1.56	21 ± 1.13	19 ± 1.12	20 ± 1.77	18 ± 0.58	15 ± 0.52	13 ± 1.77	15 ± 2.25
*P. mirabilis*	21 ± 1.72	24 ± 1.52	27 ± 1.56	17 ± 1.72	23 ± 0.77	23 ± 2.72	21 ± 0.56	21 ± 1.52	21 ± 2.21	16 ± 1.56	19 ± 0.52	16 ± 2.12
*P. aeruginosa*	21 ± 0	25 ± 1.77	26 ± 1.12	15 ± 1.12	24 ± 0.56	24 ± 2.12	21 ± 0.57	21 ± 1.15	22 ± 2.12	17 ± 1.77	21 ± 0.52	20 ± 1.77
*S. typhi*	22 ± 1	27 ± 1.12	27 ± 0.12	19 ± 2.72	21 ± 1	21 ± 2.52	20 ± 1.57	22 ± 1.56	21 ± 2.72	14 ± 0.56	16 ± 1.12	16 ± 1.52


*Bold indicated the best activity displayed by meat peptone against K. pneumoniae.*

The article "Molecular characterization of forest soil based Paenibacillus elgii and optimization of various culture conditions for its improved antimicrobial activity" was retracted in 2017. Reason: compromised peer review.

### Effect of Various Cultural Parameters on Antimicrobial Production

The various environmental parameters and cultural conditions for the production of the antimicrobial compounds by *P. elgii* have been studied on TSB + glucose + meat peptone in shaking flask condition. The present strain *P. elgii* recorded a narrow range of incubation temperature for relatively good growth and antimicrobial production. The temperature in the range of 28–30°C was found to be ideal for maximum antimicrobial compound production by *P. elgii* (**Figure 6A**). Antimicrobial activity was considerably reduced after 35°C. The best growth, as well as maximum antimicrobial compound production, was obtained at pH 7 (**Figure 6B**). Incubation period up to 7 days was found to be optimum for maximum growth as well as antimicrobial agent production by *P. elgii* (**Figure 6C**).

**FIGURE 6:** **Effect of cultural parameters on production of antimicrobial agent. (A)** p^H^, **(B)** temperature and **(C)** days. Different letters in the superscript were significantly different according to Duncan’s multiple range test (*p* < 0.05).

### Antibacterial Activity of TSB + Glucose + Meat Peptone in the Best Ideal Condition

**Table 5** showed the antibacterial activity of the crude extract of TSB + Glucose + meat peptone against test bacteria. *K. pneumonia* exhibited significant activity with a diameter of zone of inhibition of 36 mm.

**Table 5:** Antibacterial activity of crude extract from TSB + Glucose + meat peptone in the best ideal condition.

Test microbes	Zone of inhibition (mm)	
	
	Extract	Ciprofloxacin
*B. cereus*	29 ± 0.52	31 ± 0
*B. subtilis*	30 ± 1.12	33 ± 1.15
*S. aureus*	32 ± 0.77	29 ± 1.72
*S. epidermis*	31 ± 1.24	28 ± 1.52
*S. simulans*	28 ± 1	27 ± 1.52
*E. coli*	33 ± 0.57	29 ± 0
*K. pneumoniae*	36 ± 1.52	30 ± 1.75
*P. mirabilis*	32 ± 0.77	31 ± 0
*P. aeruginosa*	29 ± 1.72	32 ± 1.12
*S. typhi*	34 ± 1.72	31 ± 1.12


The article "Molecular characterization of forest soil based Paenibacillus elgii and optimization of various culture conditions for its improved antimicrobial activity" was retracted in 2017. Reason: compromised peer review.

## Discussion

For several years, actinomycetes have been productive sources of novel antimicrobial molecules (Nguyen et al., 2008; Ridley et al., 2008). Only recently, bacteria from other taxonomic groups arise as a practical novel source for various bioactive compounds with antimicrobial property and numerous successful efforts have been made in this field (Zhang et al., 2006; Wright and Sutherland, 2007; Blunt et al., 2009). In the present study, new soil bacterium exhibiting broad spectrum antimicrobial activity against various pathogens was subjected to 16S rRNA sequence screening to include the well-documented antimicrobial producers and identified as *P. elgii*.

The genus *Paenibacillus* was well-defined in 1993 after an extensive comparative investigation of 16S rRNA gene sequences of more than 51 species of the genus *Bacillus* (Ash et al., 1993). One of the enthralling characteristics of *Paenibacilli* is that some species of this genus are Gram-negative or Gram-variable although the Gram-positive dominate, consistent with their *Bacillus* originality (Elo et al., 2001; Rodriguez-Diaz et al., 2005; Roux et al., 2008). Diverse *Paenibacillus* species are well found in soil and rhizosphere region of plants. Several *Paenibacillus* species have been reported as potential biological control agents as they can produce a wide range of potent antimicrobial compounds. For example, *Paenibacillus polymyxa* E681, a plant growth-promoting (PGPR) rhizobacterium, which can successfully control the pre-emergence and post-emergence damping off diseases on sesame plants (Ryu et al., 2006). Production of antimicrobial compound has been considered as one of the chief mechanisms of plant diseases control with living microorganisms. So far, several *Paenibacillus* species have been reported to produce many antimicrobial agents with a wide spectrum inhibition of various human pathogenic bacteria and fungi (Li et al., 2007). In the present study, *P. elgii* displayed inhibitory activity against a number of Gram-positive and negative bacteria and also recorded significant antifungal activity against medically and agriculturally important fungi except *C. albicans*. *C. albicans* usually grow in biofilm matrix linked to β-1,3 glucan and exhibit a β-1,3 glucan matrix associated drug resistance mechanism against various antifungal drugs (Mitchell et al., 2013). This may be the reason for the absence of activity by *P. elgii* against *C. albicans.*

The investigation on the enhanced production of antimicrobial compounds usually involves an exploration for a appropriate fermentation medium. Fermentation media were reported to have a great influence on antimicrobial metabolite production by microorganisms (Vijayakumari et al., 2013). In our study, out of three standard fermentation media used, TSB medium recorded significant antimicrobial activity. The results of the present study clearly indicated that medium composition play a significant role in the antimicrobial secondary metabolite production by bacteria. Carbon and nitrogen sources in the fermentation media were reported to have a profound influence on the production of secondary metabolite by the microorganism (Narayana and Vijayalakshmi, 2008; Kumar et al., 2012). During our fermentation studies with different carbon sources, glucose was easily assimilated and resulted in a rapid growth for *P. elgii*. The results agreed with other *Paenibacillus* including *Paenibacillus polymyxa* RNC-D (Serrano et al., 2012). Nevertheless, glucose was reported to be a repressor of secondary metabolisms (Demain, 1999). This may be because most of the carbons were utilized rapidly for the synthesis of cellular material and little would be available for antibiotic synthesis (Pandey et al., 2005). But Kumar et al. (2013) reported fructose as the best carbon source among the water-soluble carbon sources like glucose, maltose, glycerol, mannitol, and sucrose for antimicrobial metabolite production by a *Bacillus* sp. Considering the various carbon source, simple carbon sources such as glucose, fructose, and sucrose can enhanced growth as well as bioactive metabolite production rather than more complex carbons (Calvo et al., 2002). The nature of the nitrogen source used has a notable effect on the production of the antimicrobial metabolite by the bacterium. In our study yeast extract recorded the significant effect on the antimicrobial production followed by meat peptone and beef extract. Depending on the biosynthetic pathways involved, nitrogen sources may significantly affect antibiotic formation (Gesheva et al., 2005). The results of the present study showed the requirement of the antimicrobial agent synthesis on the various medium constituents. In fact, it has been also recorded that the nature of carbon as well as nitrogen sources strongly affects antibiotic production by various microorganisms (Vilches et al., 1990). It was clear from the present study that the production of antimicrobial agents by *P. elgii* was absolutely affected by the nature and type of carbon and nitrogen sources used in the fermentation medium. The present results also recorded that antimicrobial compound production was higher in fermentation medium having glucose and meat peptone as carbon and nitrogen source, respectively.

The article "Molecular characterization of forest soil based Paenibacillus elgii and optimization of various culture conditions for its improved antimicrobial activity" was retracted in 2017. Reason: compromised peer review.

Environmental factors such as pH and temperature are acknowledged to have a thoughtful influence on growth and antibiotic production in various bacterial species (Vijayakumari et al., 2013). The changes in external pH of fermentation medium affect several cellular processes of microorganism such as regulation and biosynthesis of secondary metabolites (Sole et al., 1997). The pH of 6.5–7.5 and temperature of 25–30°C was reported to be the optimum for antibiotic production by *Bacillus* sp. (Vijayakumari et al., 2013). The *P. elgii* showed a narrow range of pH 7 for relatively good growth and antimicrobial agent production. The maximum growth, as well as highest antimicrobial activity by *P. elgii*, was achieved at pH 7 during the production of antimicrobial agent drastically reduced before and after pH 6 and 8. There are reports concerning the role of medium pH in the production of the bioactive metabolite especially antibiotics by microorganisms (Guimaraes et al., 2004). The *P. elgii* presented a narrow range of incubation temperature for comparatively good growth and antimicrobial compound production. Maximum antimicrobial compound production was obtained at 28–30°C. The temperature range satisfactory for the enhanced secondary metabolites production is usually narrow, for example, 5–10°C (Iwai and Omura, 1982). Incubation period up to 7 days was found to be significant for antimicrobial compound production by *P. elgii* and highest production was recorded at third day. These results clearly indicated that various environmental factors and cultural conditions like incubation temperature, pH and incubation period were found to have a thoughtful impact on antimicrobial compound production by *P. elgii*. In our study also TSB supplemented with glucose and meat peptone with pH 7 and incubated at 30°C for 3 days were the optimal condition for antimicrobial metabolite production by *P. elgii*.

## Conclusion

In the present study, *P. elgii* isolated from the forest soil of Wayanad, Kerala, India recorded prominent broad spectrum activity against many medically important microbial pathogens. TSB supplemented with glucose and meat peptone with pH 7 and incubated at 30°C for 3 days were the optimal condition for the enhanced antimicrobial metabolite production by *P. elgii*.

## Conflict of Interest Statement

The authors declare that the research was conducted in the absence of any commercial or financial relationships that could be construed as a potential conflict of interest.
